The article "The Change of Left Ventricular Function in Rats with Subclinical Hypothyroid and the Effects of Thyroxine Replacement" was published in 2018. Journal: Int J Endocrinol.

# The Change of Left Ventricular Function in Rats with Subclinical Hypothyroid and the Effects of Thyroxine Replacement

**DOI:** 10.1155/2018/8682765

**Published:** 2018-03-04

**Authors:** Xuedi Chen, Cuixia Gao, Ningning Gong, Yu Wang, Limin Tian

**Affiliations:** ^1^Department of Endocrinology, Gansu Provincial Hospital, Lanzhou, China; ^2^Ningxia Medical University, Yinchuan, China; ^3^Department of Ultrasonic Diagnosis, Gansu Provincial Hospital, Lanzhou, China; ^4^Gansu University of Chinese Tradition Medicine, Lanzhou, China

## Abstract

**Objective:**

The main purpose of this study was to explore the relationships between serca2a, Ryr2, adipokines, and the left ventricular function in the subclinical hypothyroidism with different TSH levels and to determine the impact of L-T4 treatment on these indexes.

**Methods:**

Sixty-five male Wistar rats were randomly divided into five groups: control group; sHT A, B, and C group; and sHT + T4 group. The sHT rats were induced by methimazole (MMI), and the sHT + T4 rats were administered with L-T4 treatment after 8 weeks of MMI administration. Serum TT4, TSH, APN, chemerin, and TNF-*α* were detected by radioimmunoassay kits and ELISA kits; left ventricular function was measured by PowerLab system via subclavian artery catheter. The expression of Serca2a, Ryr2, APN, chemerin, and TNF-*α* were detected by RT-PCR, Western blot, and immunohistochemistry.

**Results:**

The sHT groups had significantly higher TSH, chemerin, and TNF-*α* and lower Serca2a, Ryr2, and APN. The left ventricular pressure and heart rate in sHT groups were significantly lower in control and sHT + T4 group. Histopathological examination revealed the pathological changes in the sHT rats' heart. L-T4 administration reduced TSH level and improved left ventricular function.

**Conclusions:**

TSH can impair left ventricular function by regulating several factors, and L-T4 treatment ameliorates it in sHT rats.

## 1. Introduction

Subclinical hypothyroidism (sHT) is a common thyroid dysfunction, which has a milder thyroid-stimulating hormone (TSH) and a normal range of serum thyroid hormone level [1]. It is generally known that TSH is one of the important factors of cardiovascular disease in sHT, and increasing studies show that dysfunction of cardiac systolic and diastolic is the common abnormality in sHT [2, 3], especially left ventricular diastolic function impaired. Previous studies demonstrate that sarcoplasmic/endoplasmic reticulum Ca2 + ATPase 2a (Serca2a) and ryanodine receptor (Ryr2) have significant roles for abnormalities of cardiac systolic and diastolic functions [4], but these changes in sHT with different TSH levels are still unclear. Besides, adipokines also impact left ventricular function to a certain degree, but the relationships between them and sHT are still dim.

The article "The Change of Left Ventricular Function in Rats with Subclinical Hypothyroid and the Effects of Thyroxine Replacement" was published in 2018. Journal: Int J Endocrinol.

Cardiac muscle is an important target tissue of TSH, and TSH plays an important role in cardiac function abnormalities, which is regulated highly by binding to TSH receptor. Our previous study found that the Serca2a activity can be inhibited by prolonged exposure to elevated TSH levels by binding to TSHR [5] and the changes independent of thyroid hormone, but which hardly represent physiological status in vivo. Besides, whether and how change of Ryr2 in sHT remains controversial. So, Serca2a and Ryr2's activity and expression are worth studying in sHT.

In numerous regulating cardiac function factors, adipokines have always taken an important status. Likewise, TSH stimulates the production of adipokines in human abdominal adipose tissue by applied functional TSH receptor protein [6]. In addition, a study had found that a portion of adipokines was expressed to a certain amount in the heart [7]. However, whether these expressions regulated by TSH and what kind of relationship exists between adipokines and the left ventricular function in sHT lacked reference researches.

Adiponectin (APN) is a pivotal hormone secreted by adipocytes which present an inverse proportion to the degree of obesity and insulin resistance [8]. Many researches [9, 10] show the potential involvement of APN in improving cardiovascular function, and low dose of APN may be a risk factor in congestive heart failure (CHF). Besides, a recent study found that APN was exhibited significantly in high serum levels in hyperthyroid patients [11], but the study of the relationship between APN and TSH was not fully studied yet. Tumor necrosis factor-alpha (TNF-*α*) is a proinflammatory cytokine secreted by the cardiomyocytes. Previous studies had verified that TNF-*α* performed a restraining function in cardiac muscle contraction and stretch [12, 13]. The experiments of an intact heart found that a low concentration of TNF-*α* acted on the intact heart produced negative inotropic effects [14]. In recent years, increasing studies show that thyroid dysfunction is related to TNF-*α* [15]. Chemerin was initially found and expressed at the highest levels in white adipose tissues. Goralski et al. proved chemerin mRNA was expressed to a certain amount in the heart [7], and a study showed that plasma chemerin concentrations were increased in dilated cardiomyopathy (DCM) [16]. However, researches that explore the changes of adipokines have been very limited in sHT and the effect of L-T4 treatment [17].

The relationships between serca2a, Ryr2, adipokines, and the left ventricular function in the sHT with different TSH levels have not yet been investigated. It is also not fully clear the effect of levothyroxine (L-T4) treatment on left ventricular function and these factors. Our study aims to observe the relationships of left ventricular function and these factors in sHT rats and to determine the impact of L-T4 treatment on these indexes.

The article "The Change of Left Ventricular Function in Rats with Subclinical Hypothyroid and the Effects of Thyroxine Replacement" was published in 2018. Journal: Int J Endocrinol.

## 2. Materials and Methods

### 2.1. Modeling Stage

Sixty-five male SPF Wistar rats weighing 160–180 g were purchased from the University of Gansu Traditional Chinese Medicine Experimental Animal Center (Lanzhou, Gansu, China) and fed in a specific pathogen-free (SPF) animal laboratory. The rats were randomly divided into four groups after a period of environmental adaptation (7 days): control group (*n* = 10), sHT A group (*n* = 15), sHT B group (*n* = 15), and sHT C group (*n* = 25). 5 mg·kg^−1^·d^−1^ [18], 15 mg·kg^−1^·d^−1^, and 20 mg·kg^−1^·d^−1^ methimazole (MMI) were gavaged, respectively, to rats in sHT A, B, and C groups. Control group rats were administered with 10 ml·kg^−1^·d^−1^ saline. Serum thyroid hormone and TSH levels were measured every two weeks to verify the success of the induction of subclinical hypothyroidism in the experimental groups. After 8 weeks, we detected that levels of TSH increased in the sHT C group rats, compared with the control group rats, and levels of TT4 unchanged. The sHT rat models in the sHT C group were successful. Then, we randomly selected ten rats from the sHT C group for adding L-T4 administration of 6 *μ*g·kg^−1^·d^−1^ [19], which named the sHT + T4 group (*n* = 10), and we continued giving the sHT + T4 group 20 mg·kg^−1^·d^−1^ MMI. In this pried, sHT groups' rats were continually gavaged with a corresponding dose of MMI. During the experiment, body weight was measured weekly. Serum thyroid hormone and TSH levels were measured every two weeks to assess the thyroid function.

### 2.2. Drugs and Doses

MMI (Sigma Chemical, MO, USA) and L-T4 (Merck KGaA DE-MRK) was dissolved in physiological saline, and the doses of the abovementioned have been tested in a four months preexperiment.

### 2.3. Hemodynamic Parameters

The rats were performed under 10% chloral hydrate (3 ml/kg i.p.) anesthesias. The catheter was inserted in the left ventricle via the subclavian artery for the assessment of LV function. After the catheter entering the left ventricle, the ventricular pressures and heart rate were registered. During measurements, rats physiologically breathed without mechanical ventilation. All of the signals were recorded and analyzed using a PowerLab system and software (AD Instruments, Dunedin, New Zealand) [20].

### 2.4. Biochemical Measurements

Serum concentrations of TT4 and TSH were detected using radioimmunoassay kits (Beijing North Institute of Biological Technology Co., Ltd, Beijing, China). APN, chemerin, and TNF-*α* were detected by ELISA kits (Enzyme-linked Biotechnology Co., Ltd, Shanghai, China).

The article "The Change of Left Ventricular Function in Rats with Subclinical Hypothyroid and the Effects of Thyroxine Replacement" was published in 2018. Journal: Int J Endocrinol.

### 2.5. Quantitative RT-PCR

#### 2.5.1. Reverse Transcription

Total RNAs were isolated from myocardial tissue samples of rats using TRIzol reagent according to the manufacturer's instruction (Invitrogen, USA). After being isolated, the RNA was reverse-transcribed to cDNA with the use of a 5x PrimeScript® RT Master Mix Kit (TaKaRa, Dalian, China). For the reverse transcription, the following protocol was used: 2 *μ*l RT Master Mix, 500 ng total RNA, and RNase-free dH_2_O up to 10 *μ*l (a reaction volume of 10 *μ*l is the highest value to accommodate 500 ng RNA samples according to the manufacturer's instructions). The mass of total RNA was detected by Ultraviolet Spectrophotometer (Thermo Fisher Scientific, MA, USA). The reverse transcription reaction consisted of 15 minutes of reaction: 37°C for 15 minutes and 85°C for 5 seconds using the iCycle system (Bio-Rad, CA, USA).

#### 2.5.2. Polymerase Chain Reaction

For detection, the following reagents were used: 12.5 *μ*l SYBR® Premix EX TaqTM II (TaKaRa, Dalian, China), 1 *μ*l of each receptor-specific forward primer, 1 *μ*l of each receptor-specific reverse primer, 2 *μ*l^∗^2 cDNA, and 8.5 *μ*l dH2O. The PCR reaction consisted three stages: stage 1, 95°C for 30 seconds; stage 2, 95°C for 5 seconds and 60°C for 30 seconds followed by 40 cycles; stage 3, dissociation. The whole detecting process used the FTC3000 PCR System (Funglyn Biotech, Canada). Relative mRNA expression was calculated using the 2^−ΔΔCt^ method. We used the expression of housekeeping gene glyceraldehyde-3-phosphate dehydrogenase (GAPDH) to normalize mRNA expression (Table 1).

#### 2.5.3. Western Blot

In the process of protein extraction, the fragment of the tissue was broken in the RIPA Lysis buffer (according to the manufacturer's instructions, 1 ml buffer was added in 100 mg tissue). The tissue cocktail was homogenized by electrically driven Tissue Homogenizer (IKA, Germany). Subsequently, protein concentration was determined using a BCA Protein Assay Kit (Solarbio Bioscience & Technology Co., LTD, Beijing, China). For the Western blot analysis, 10 *μ*l samples (~50 *μ*g protein) were separated by 8% SDS-PAGE (Solarbio Bioscience & Technology Co., LTD, Beijing, China) and transferred to PVDF membranes. After being transferred, the membranes were blocked at 5% nonfat milk for 2.5 h at ambient temperature and then incubated with the following antibodies overnight at 4°C: Serca2a (Abcam, Cambridge, UK) (1 : 1000), Ryr2 (GeneCreate Co., Ltd, Wuhan, Chain) (1 : 500), chemerin (Abcam, Cambridge, UK), adiponectin (Abcam, Cambridge, UK) (1 : 1000), TNF-*α* (ImmunoWay Biotechnology Company Biotechnology Co., USA) (1 : 200), and GAPDH (ImmunoWay Biotechnology Company Biotechnology Co., USA) (1 : 1000). After incubated with first antibodies, the membranes were then incubated with a secondary antibody for 2 h at room temperature. The specific protein bands were visualized using ECL-Plus Western blot detection reagents (ImmunoWay Biotechnology Company Biotechnology Co., USA). Densitometric analysis of band intensity was completed using Quantity-One software (Bio-Rad, CA, USA).

The article "The Change of Left Ventricular Function in Rats with Subclinical Hypothyroid and the Effects of Thyroxine Replacement" was published in 2018. Journal: Int J Endocrinol.

### 2.6. Histopathology of the Heart

In this part, the five group rats were sacrificed under anesthesia and the hearts were used for histopathological study at the end of modeling. The hearts were isolated and soaked in 10% paraformaldehyde phosphate buffer solution. After 2-3 days, the hearts were prepared for routine paraffin sections and dehydrated, passing through different concentration of alcohol and embedded sections in paraffin blocks. The sections were separated by 20 *μ*m to obtain approximately random sections for morphometric measurements. Hematoxylin and eosin were used for staining. Normal deparaffinized heart tissue was prepared for immunohistochemistry. We used 10 mM sodium citrate (pH 6.0) buffer to expose target proteins and retrieve antigen by microwaving for 8–15 minutes. Retrieval tissues were soaked in 3% BSA-PBS at 25°C for 30 minutes and then, respectively, bonded at SRECA2a (Abcam, Cambridge, UK) (1 : 200), Ryr2 (GeneCreate Co., Ltd, Wuhan Chain) (1 : 200), chemerin (Abcam, Cambridge, UK) (1 : 200), adiponectin (Abcam, Cambridge, UK) (1 : 100), and TNF-*α* (ImmunoWay Biotechnology Company Biotechnology Co., USA) (1 : 200) for overnight at 4°C. The negative tissue control groups were bonded at PBS instead of the first antibody for overnight at 4°C.Then the slides were washed with phosphate buffer and incubated with the secondary antibody. Then the slides were stained by DAB.

## 3. Ethics Statement

This study was strictly launched according to the Care and Use of Laboratory Animals by the National Institutes of Health. The program has been approved by the Committee on the Ethics of Animal Experiments of the College of Gansu Traditional Chinese Medicine Experimental Animal Center (permit number: SYXK 2011–0001).

## 4. Statistics

Data are expressed as mean ± SD. A *p* value of <0.05 was considered significant. One-way analysis of variance (ANOVA) was conducted for statistical analysis using SPSS 17.0 software (SPSS Inc., Chicago, IL, USA). Analyses using Pearson correlations were conducted to examine the relationships of TSH and Serca2a, Ryr2, APN, chemerin, and TNF-*α*.

The article "The Change of Left Ventricular Function in Rats with Subclinical Hypothyroid and the Effects of Thyroxine Replacement" was published in 2018. Journal: Int J Endocrinol.

## 5. Results

### 5.1. Physiological Status

During the molding stage, mores serious depilation occurrred in sHT rats with increasing dose of MMI. We found that the ability of resisting catch in sHT rats was weaker than control rats, which was the same with previous studies [21, 22]. We also found that the sHT rats experienced a stunted growth pattern compared with the control rats, and L-T4 treatment improved the body weights of sHT rats (Figure 1).

### 5.2. Serum Index Levels

There were no significant differences in the serum TT4 between each group. The serum TSH level in the sHT groups (A, B, and C) was significantly increased compared with that in the control group (*p* < 0.05). In the sHT + T4 group, the serum TSH level was statistically decreased compared with the sHT C group (*p* < 0.05) but still increased compared with the control group (*p* < 0.05). Alterations in increased serum levels of chemerin and TNF-*α* in sHT A, B, and C coincided with the trend of TSH, and L-T4 treatment could decrease these changes in the sHT + T4 group. But analysis of serum APN levels has an opposite result (Table 2). Pearson correlation showed a positive correlation between chemerin, TNF-*α*, and TSH(*r* = 0.858, *p* < 0.01; *r* = 0.876, *p* < 0.01). A negative correlation was found between APN and TSH (*r* = −0.868, *p* < 0.01).

### 5.3. Hemodynamic Data

Every parameter hemodynamic was improved via L-T4 treatment but did not catch the standard of normal control. As shown in Table 3, the sHT rats had a significant decrease in ventricular pressure and HR compared with the control group rats. The L-T4 treatment rats had higher ventricular pressure and HR compared with the other group rats (Table 3). Pearson correlation showed a negative correlations which were found between TSH and LVSP (*r* = −0.706, *p* < 0.01), LVEDP (*r* = −0.857, *p* < 0.01), MP (*r* = −0.841, *p* < 0.01), and HR(*r* = −0.855, *p* < 0.01).

### 5.4. The Expression of Ryr2, Serca2a, and Adipocytokines

As Figure 2 shows us, the expressions of Serca2a and Ryr2 were decreased in sHT rats compared with the control rats. We also found that the expression of Serca2a and Ryr2 was improved by L-T4 treatment. The most important information offered to us was that Ryr2 and Serca2a activity decreased concentration dependently. Compared with the control group, the activity of Ryr2 and Serca2a decreased by 29.34% and 30% in the sHT A group (^∗^*p* < 0.05), decreased by 67.18% and 53.64% in the sHT B group (^∗∗^*p* < 0.001), and decreased by 78.31% and 68.57% in the sHT C group (^∗∗^*p* < 0.001). APN decreased in sHT A groups (^∗^*p* < 0.05) and sHT B and C groups (^∗∗^*p* < 0.001) but increased in the sHT + T4 group compared with the control group. Chemerin and TNF-*α* have increased in sHT A groups compared with the control group (^∗^*p* < 0.05) and sHT B and C groups (^∗∗^*p* < 0.001), and L-T4 treatment downregulated these levels (Figure 2). Pearson correlation showed a negative correlation between Ryr2, Serca2a, APN, and TSH (*r* = −0.814, *p* < 0.01; *r* = −0.753, *p* < 0.01; *r* = −0.69, *p* < 0.001). Positive correlations were found between chemerin, TNF-*α*, and TSH (*r* = 0.637, *p* < 0.001; *r* = 0.709, *p* < 0.001).

The article "The Change of Left Ventricular Function in Rats with Subclinical Hypothyroid and the Effects of Thyroxine Replacement" was published in 2018. Journal: Int J Endocrinol.

The expression of protein serca2a, Ryr2, and APN was decreased in the sHT A, B, and C groups, and LT-4 treatment improved the expression of them. The protein of chemerin and TNF-*α* presents a gradually increasing trend from the control group to the sHT C group, and LT-4 treatment decreased them. GAPDH was used as an internal reference. Histogram reflected an approximate variation trend of protein, and GAPDH as an internal reference was used in calculating the expression of protein (Figure 3).

In HE staining, myocardial fibers of rats in the control group were arranged regularly and contacted closely with cell space and the nuclear chromatin toward the center with the even distribution. But the structure of the cardiac muscle of rats in the sHT C group was loose and has a disordered arrangement. Some cardiac cells got swelling and plasma cell infiltration could be observed in cell space. In sHT A and B groups, those changes were relatively better than that in the sHT C group. In the sHT + T4 group, morphological changes of myocardial cells were better than those in sHT groups, especially better than high serum TSH groups. In other words, L-T4 treatment ameliorated the above impairment in the sHT + T4 group (Figure 4).

In immunohistochemical staining, the positive areas are dyed in brown (the pointed arrow). The positive areas of Serca2a (Figure 5(a)), Ryr2 (Figure 5(b)), and APN (Figure 5(c)) were shown a decreasing trend from the control group to sHT C group, and positive areas were increased in the sHT + T4 group. The positive areas of chemerin (Figure 5(d)) and TNF-*α* (Figure 5(e)) were shown an increasing trend from the control group to the sHT C group and which were decreased in the sHT + T4 group. PBS was used in immunohistochemical staining instead of first antibody as negative tissue comparison.

## 6. Discussion

An innovation of the study is the establishment of statistically different serum TSH levels in sHT rat groups. According to Santi et al. [18], different doses of MMI in establishing the sHT rat model had been verified and adjusted in a 4-month preexperiment before starting the experiment. The sHT rat model with 20 mg·kg^−1^·d^−1^ of MMI was successfully established after 8 weeks. The sHT rat model with 5 mg·kg^−1^·d^−1^ and 15 mg·kg^−1^·d^−1^ of MMI was established, respectively, at 16 weeks and 13 weeks. Long time experiment benefits us to investigate the effects of different levels of TSH and the treatment of L-T4 on left ventricular function and adipokines.

The article "The Change of Left Ventricular Function in Rats with Subclinical Hypothyroid and the Effects of Thyroxine Replacement" was published in 2018. Journal: Int J Endocrinol.

The change of left ventricular function in sHT has always taken the attention in clinical trials. Recent clinical trials have shown an impaired left ventricular diastolic function in sHT patients [2], and Sunbul et al. described in a study that untreated patients with sHT were associated with impairment in left ventricular longitudinal myocardial function [23]. However, a previous study with a number of subjects in sHT found lower parameters in left ventricular functions among sHT patients, but no statistically significant association exists between them [24]. Here, our study shows that LVSP, LVEDP, and HR decreased in the sHT rat group, and negative correlations were found between TSH and this index, with the present study [25]. This heterogeneity mainly came from the difference of serum TSH levels and sample size.

During the left ventricular diastole stage, the activity of the sarcoplasmic reticulum calcium ATPase (Serca2a) is crucially important [26]. Ryr2 is the most important Ca^2+^ release channel in the sarcoplasmic reticulum and plays a vital role in systolic stage [27, 28]. In our research, we observed that expression of the mRNA and protein of Serca2a and Ryr2 was downregulated by serum TSH in sHT rats, and this downregulation is a kind of concentration-dependent relationship with TSH. These demonstrated that in the sHT state a relatively elevated concentration of serum TSH may lead to more severe systolic and diastolic dysfunction by impacting Serca2a and Ryr2 activities compared with relatively low TSH level in sHT, which is similar with our previous study [5]. Here, we first simultaneously investigated left ventricular function both systolic and diastolic aspects and found that gradually raised serum TSH levels not only accelerated the progression of the illness from sHT to hypothyroidism but also aggravated in damaging the left ventricular function both in the systolic and diastolic stage.

We further demonstrated APN expressed in cardiac muscular tissue and also found APN was downregulated in sHT rats' hearts and a negative correlation between it and TSH. Before our study, Yildiz et al. found a negative correlation of TSH levels and APN in women with sHT [29], which is similar to our results. However, another study showed that there was no correlation between serum APN and TSH [30]. We analyzed the conflict and found that the main reasons may be as follows: (a) our study directly detected the expression of APN in sHT rats' heart, which only reflects the expression levels of APN in cardiac muscular tissue; (b) the difference of sample size, serum APN, and TSH levels could also affect the results. Researches demonstrate that APN regulates cardiac function and the mainstream view is that APN improves the left ventricular function and prevents further deterioration in it [9, 10, 31]. In our study, the expression of APN in cardiac muscular tissue was decreased with left ventricular function impairment. But the mechanism of this special correlation has not been recognized clearly yet.

The article "The Change of Left Ventricular Function in Rats with Subclinical Hypothyroid and the Effects of Thyroxine Replacement" was published in 2018. Journal: Int J Endocrinol.

As a novel adipokine, chemerin regulates adipogenesis and adipocyte metabolism [32], and the expression of chemerin in experimental rats consisted in the increased of TNF-*α* [33]. Some studies reported that the baseline of chemerin and TNF-*α* level shows an increasing trend in sHT patients compared with the euthyroidism group, but there was no statistical difference between them [17, 34]. Here, we found that the levels of chemerin and TNF-*α* in sHT rats were significantly increased compared with the control rats. Moreover, the levels of chemerin and TNF-*α* positively associated with TSH. The reason may be due to the differences of TSH concentrations. In the recent years, chemerin and TNF-*α* have gradually taken focus on cardiovascular disease [35], but there is a lack of clinical studies for the changes of above adipokines in sHT. Goralski et al. described in a previous study that chemerin was expressed to a certain amount in the cardiac muscle of rats [7]. For our study, chemerin and TNF-*α* level could be detected in sHT rats and show a negative correlation with left ventricular function. These results may suggest that chemerin and TNF-*α* were involved in occurrence and development of left ventricular impairment, and the mechanism may be related to ischemia-reperfusion conditions [36] and oxidative stress [37].

The establishment of sHT + T4 rats in our study aims to investigate the effect of L-T4 replacement in left ventricular function. A recent clinical trial found that low-dose L-thyroxine may improve the left ventricular diastolic function in patients with sHT [38]. In this study, the activity of Serca2a and Ryr2 was improved with L-T4 treatment in the sHT + T4 group, and histopathological analysis revealed that morphological changes of myocardial cells in the sHT + T4 group was better than that in the sHT rat group. Hemodynamic parameters were improved in sHT + T4 group rats, which were similar to our previous study [25]. Besides, Seifi et al. reported that APN mRNA in hypothyroid rats was significantly increased after 2 weeks of L-T4 treatment [39]. Here, we observed the APN expression was increased and chemerin and TNF-*α* were significantly decreased in L-T4 treatment rats by gene and protein examination. These results suggested that some adipokines were recommended as the potential therapeutic target for ameliorating the left ventricular function in sHT.

The article "The Change of Left Ventricular Function in Rats with Subclinical Hypothyroid and the Effects of Thyroxine Replacement" was published in 2018. Journal: Int J Endocrinol.

In conclusion, our study demonstrated that left ventricular function was impaired in sHT rats through regulating the activity of serca2a, Ryr2, and some adipokines, and the high level of TSH plays a key role in this process. So, we can confirm that high TSH levels act on the cardiac muscle for a long time which could weaken the ability of myocardial systolic and diastolic function. All of these afford a reference point for clinicians to assess cardiovascular risk through detecting serum APN, chemerin, and TNF-*α* level in sHT patients with high TSH levels. Besides, L-T4 treatment has a beneficial effect for restoring cardiomyocytes and recovering the left ventricular function in the early impaired stage. Hence, clinicians treat patients who have high cardiovascular risk to reduce the rate of cardiovascular disease.

## Figures and Tables

**Figure 1:** sHT rats experienced a stunted growth pattern and L-T4 treatment improved the body weights of sHT rats.

**Figure 2:** The expression of serca2a, Ryr2, APN, chemerin, and TNF-*α* mRNA in the cardiac muscle tissue was measured with real-time PCR. ^∗∗^*p* < 0.001 and ^∗^*p* < 0.05.

**Figure 3:** The protein expression of serca2a, Ryr2, APN, chemerin, and TNF-*α* in the cardiac muscle tissue was measured with Western blot.

**Figure 4:** Representative histological sections of the cardiac muscle stained with HE (200x).

**Figure 5:** Representative histological sections of the cardiac muscle stained with immunohistochemical (400x).

**Table 1:** The sequences of the abovementioned primers.

Gene	Forward	Reverse
Rat Serca2a	5′-GGAGGCGTTGCTAAACACTC-3′	5′-GAACCAGCCTTCGATATTGG-3′
Rat Ryr2	5′-CTCAAACCACGAACACATCG-3′	5′-TCCACATCAAAGTCCTCCAA-3′
Rat APN	5′-TCACTCAGCATTCAGCGTAG-3′	5′-CTGATACTGGTCGTAGGTGAAG-3′
Rat chemerin	5′-GGAGATCGGTGTGGACAGTG-3′	5′-GGGTCCAGTTTGATGCAGG-3′
Rat TNF-*α*	5′-CCACCACGCTCTTCTGTCTAC -3′	5′-ACCACCAGTTGGTTGTCTTTG-3′
Rat GAPDH	5′-GGCACAGTCAAGGCTGAGAA-3′	5′-ATGGTGGTGAAGACGCCAGT-3′

**Table 2:** 

	Control	sHT A	sHT B	sHT C	sHT + T4
TT_4_ (ng/ml)	67.11 ± 6.86	61.09 ± 9.837	61.35 ± 9.51	60.34 ± 10.59	59.71 ± 5.93
TSH (*μ*IU/ml)	0.416 ± 0.058	0.623 ± 0.067^a^	0.729 ± 0.07^ab^	0.815 ± 0.067^abc^	0.621 ± 0.084^ad^
Chemerin (pg/ml)	202.26 ± 17.27	314.33 ± 16.99^a^	355.15 ± 17.09^ab^	365.06 ± 11.63^ab^	260.07 ± 10.79^ad^
TNF-*α* (ng/l)	143.75 ± 18.4	222.64 ± 14.13^a^	279.23 ± 12.79^ab^	288.33 ± 15.89^ab^	178.47 ± 10.29^ad^
APN (*μ*g/l)	114.69 ± 4.44	77.22 ± 3.08^a^	68.58 ± 2.92^ab^	59.45 ± 2.41^abc^	102.53 ± 3.17^ad^

^a^ *p* < 0.05 versus control group; ^b^*p* < 0.05 versus sHT A group; ^c^*p* < 0.05 versus sHT B group; ^d^*p* < 0.05 versus sHT C group.

The article "The Change of Left Ventricular Function in Rats with Subclinical Hypothyroid and the Effects of Thyroxine Replacement" was published in 2018. Journal: Int J Endocrinol.

**Table 3:** 

	Control	sHT A	sHT B	sHT C	sHT + T4
LVSP (mmHg)	123.1 ± 5.93	118.43 ± 4.31^∗#^^b^	111.53 ± 5.97^∗#^^a^	106.8 ± 3.96^∗#^^a^	115.8 ± 4.54^∗^
LVEDP (mmHg)	16.1 ± 1.66	11.67 ± 1.67^∗#^^a^	8.67 ± 1.54^∗#^^b^	5.4 ± 1.76^∗#^^a^	7.9 ± 1.66^∗^
MP (mmHg)	51.77 ± 2.77	47.38 ± 1.82^∗#^^a^	42.96 ± 2^∗#^^b^	39.2 ± 1.89^∗#^^a^	43.87 ± 1.95^∗^
HR (beats/min)	405.8 ± 15.19	358.53 ± 18.19^∗#^^a^	322.87 ± 10.45^∗#^^b^	299.8 ± 9.95^∗#^^a^	332 ± 12.95^∗^

Compared with the control group; ^∗^*p* < 0.05. sHT A, B, and C compared with each other; ^#^*p* < 0.05. LVSP: sHT B and sHT C compared with sHT + T4 group; *p* < 0.05. sHT A compared with sHT + T4 group; ^b^*p* > 0.05. LVEDP, MP, and HR: sHT A and sHT C compared with sHT + T4 group; ^a^*p* < 0.001. sHT B compared with the sHT + T4 group; ^b^*p* > 0.05. LVSP: left ventricular systolic pressure; LVEDP: left ventricular end diastolic pressure; MP: mean pressure; HR: heart rate.

## Additional Points

*Limitations*. The research has several limitations. First, although hemodynamic parameters could reflect the assessment of cardiac function in rats, the measurement of invasive detection can only be permitted in animals. Second, our research was limited to male rats, which restricts our results. Third, the results of Western blot and RT-PCR only represent several rats, and the results have limitation from measurement. So, vitro experiment may be worth to implement in future.
